RETRACTED

# Biologically Synthesized Peptides Show Remarkable Inhibition Activity against Angiotensin-Converting Enzyme: A Promising Approach for Peptide Development against Autoimmune Diseases

**DOI:** 10.1155/2022/2396192

**Published:** 2022-06-20

**Authors:** Nosheen Mujtaba, Nazish Jahan, Adil Jamal, Shazia Abrar, Shumaila Kiran, Atizaz Rasool, Md Belal Hossain, Fayez Saeed Bahwerth, Ibtesam Nomani, Khalid Javed Iqbal

**Affiliations:** ^1^Department of Chemistry, Faculty of Sciences, University of Agriculture, Faisalabad, Pakistan; ^2^College of Nursing, Umm Al Qura University, Makkah-715, Saudi Arabia; ^3^Department of Applied Chemistry, Government College University, Faisalabad, Pakistan; ^4^Department of Plant Pathology, Faculty of Agriculture, Sher-e-Bangla Agricultural University, Sher-e-Bangla Nagar, Dhaka-1207, Bangladesh; ^5^Central Laboratory and Blood Bank, King Faisal Hospital, Makkah-24235, Saudi Arabia; ^6^Department of Zoology, The Islamia University of Bahawalpur, Bahawalpur, Pakistan

## Abstract

Angiotensin-converting enzyme (ACE) regulates several biological functions besides its vital role in immune functions. ACE is elevated in immune cells in inflammatory diseases including atherosclerosis, granuloma, chronic kidney disease, and also autoimmune diseases, like multiple sclerosis, rheumatoid arthritis, and type I diabetes. No significant information prevails in the literature regarding the isolation, identification, and profiling of potential ACE inhibitory peptides. In the present study, indigenous crop varieties like seeds (peanut, corn, oat, sunflower, chickpea, parsley, cottonseed, papaya, sesame, and flaxseed) were used to evaluate their ACE inhibition activity. Variables including hydrolysis time, enzyme-to-substrate ratio (E/S), pH, and temperature were standardized to acquire the most suitable and optimum ACE inhibition activity. Seeds of cotton, chickpea, and peanuts displayed remarkably maximum ACE inhibition activity than other plants. The study disclosed that maximum ACE inhibitory activity (86%) was evaluated from cottonseed at pH 8.0, temperature of 45°C, hydrolysis time of 2 hrs, and enzyme to the substrate (E/S) ratio of 1 : 5 followed by peanuts (76%) and chickpea (55%). SDS-PAGE confirmed that vicilin protein is present in cottonseed and peanut seed while cruciferin and napin proteins are present in chickpeas. LC-MS/MS analysis disclosed potential novel peptides in hydrolyzed cottonseed that can be ascribed as potential ACE inhibitors which have never been reported and studied earlier. The current study further showed that cottonseed peptides due to their promising ACE inhibitory activity can be a valuable source in the field of ACE inhibitor development.

RETRACTED

## 1. Introduction

Angiotensin-converting enzyme (ACE) is involved in inflammation and in the stimulation of T-cells by certain antigenic peptides. In autoimmune disorders, ACE levels are increased. Certain immune functions are suppressed and inflammatory or autoimmune diseases are inhibited by ACE inhibitors [1]. Autoimmune disease treatments minimize symptoms while suppressing the immune system. Most autoimmune disorders are inflammatory, involving T-cell responses and cytokine production [2]. Hence, as a result, biologics-based targeted therapies are designed to target specific proteins and protein-protein interactions. Peptides and peptidomimetics are being developed with the goal of binding to these proteins and modulating the immune system. Several costimulatory substances that are involved in inflammation and the T-cell response have been identified as potential targets for the treatment of autoimmune diseases [3]. Additionally, with the rise in autoimmune diseases (type 1 diabetes, rheumatoid arthritis, lupus, psoriasis, celiac disease, etc.), the use of multifunctional immunomodulatory peptides and/or anti-inflammatory and antimicrobial peptides in vaccines has gained importance [4–6].

Peptides and peptidomimetics can act as immunomodulators by either blocking or stimulating the immune response to generate tolerance. The study of peptide synthesis and modified amino acid side chains has led to a new class of autoimmune therapeutic drugs [7]. Peptides combine the benefits of tiny molecules with proteins [8]. However, peptides have limited in vivo enzymatic stability, short half-life, and rapid renal elimination [9]. The design of peptides/peptidomimetics for immunomodulation in autoimmune diseases such as HIV infection, rheumatoid arthritis, multiple sclerosis, and systemic lupus is of prime importance.

The discovery of plant primary metabolites such as proteins and peptides for disease management has ushered in a new era for the development of plant-based peptides as therapeutic candidates [10]. Bioactive peptides have been found in abundance in both animal and plant sources. Plants possess different ACE inhibitory peptides which can be obtained by enzymatic hydrolysis [11, 12]. The peanut, cottonseed, and chickpea are not only the most important crops broadly used as nutrient sources for animals and humans, but they also possess natural ACE inhibitory activity [13]. Plant peptides are still being investigated, and just a few bioactive peptides have been found in soy, wheat, and other plants [14]. Proteins have high-fat content in animals and can cause diseases such as hypertension and cardiac disease if consumed in large quantities. Plant proteins, on the other hand, have no associated fat and no side effects [15].

RETRACTED

To the best of our knowledge and information available, no significant literature prevails regarding the screening and development of inhibitory peptides and their role in autoimmune diseases. Therefore, the aim of the present research was to evaluate the ACE inhibition potential of indigenous plants for the production of inhibitory peptides. Our study focused on the screening of plants for their ACE inhibition activity. This study also is aimed at development of potential ACE peptide inhibitors from plants and protein profiling using the liquid chromatography mass spectrometry (LC-MS/MS) approach. These identified potential ACE inhibitory peptides from plants can be used as a source in the development of antihypertensive drugs in the pharmaceutical field in the future to cure autoimmune diseases/disorders.

## 2. Material and Methods

### 2.1. Preparation of Crude Extracts

The seeds of local varieties used in this study were obtained from the Seed section of Ayyub Agriculture Research Institute (AARI), Faisalabad, Punjab, Pakistan. A fine powdered seed of each plant was mixed with distilled water thoroughly for 2 hrs until the mixture was homogenized. The extract was filtered through Whatman No. 1 filter paper, and the solvent was evaporated with a rotary evaporator. Extracts were stored at -20°C for further analysis.

### 2.2. Extraction of Angiotensin-Converting Enzyme (ACE)

ACE extracted from rabbit lung powder was used as reported earlier with minor modifications [16]. Freshly slaughtered healthy rabbit lungs were washed thoroughly with saline solution (0.8%) and pulverized later using phosphate-buffered saline (PBS). The pulverized tissue was centrifuged at 4000 g for 15 min. The supernatant was discarded, and the centrifuged sample was washed with acetone for 3-4 times followed by continuous stirring. Acetone was dissolved in phosphate buffer (pH 8.3). The sample was stirred for 10 hrs and centrifuged at 4000 g for 45 min at room temperature. Centrifuged samples were further proceeded for ACE extraction [17, 18]. The drug captopril was used as a positive control (1 mg/mL) [19, 20]. Captopril (25 mg) was ground to fine powder, and extract was prepared using 25 mL of deionized distilled water. The prepared extract was filtered using a Whatman filter paper.

### 2.3. Determination of ACE Inhibition Activity

The ACE inhibition activity of plants seeds was determined using the reported method [21]. To prepare 25 *μ*L of each sample solution, 60 *μ*L of Hippuryl-L-histidyl-L-leucine (5 mM) and 100 mM of sodium borate buffer (pH 8.3) having NaCl (300 mM) were mixed at 40°C for 15 minutes. The reaction was initiated by adding 10 *μ*L of ACE, and the mixture was further incubated later at 40°C for 35 min. The incubated reaction was terminated using HCl (1 M). 0.5 mL of ethyl acetate was added and centrifuged at 3000 rpm for 15 min at 4°C to extract hippuric acid (HA). Upper ethyl acetate layer (0.2 mL) was separated and was evaporated at room temperature. The resulted HA was dissolved in 1.0 mL deionized distilled water, and the optical density of this solution was calculated at 228 wavelength using a UV spectrophotometer. The ACE inhibition activity was determined by Zheng et al.'s method [22]. ACE inhibition (%) was calculated using the following formula:

ACE inhibition (%) = 100 × ([(*A* − *B*) − (*C* − *D*)]/(*A* − *B*)).(1)

*A* is the absorbance of ACE, *B* is the absorbance of the reaction blank, *C* is the absorbance in the presence of ACE and inhibitor, and *D* is the absorbance of the sample blank.

RETRACTED

All observations were carried out in triplicates, and results were expressed as the mean ± SE.

### 2.4. Preparation of Protein Isolates and Sample Digestion

The plants with higher ACE inhibition activity (>50% including peanut, chickpea and cottonseeds) were selected for protein extraction. Protein was isolated using the previously reported protocol [23]. Seeds of selected plants were ground to fine powder and defatted with *n*-hexane for 7 hours using the Soxhlet apparatus. Protein extracts (1 : 12 *w*/*v*) were prepared using NaOH (0.09 M) at room temperature. The extracts were centrifuged at 3000 rpm for 25 minutes. The higher film was standing apart, set to pH 5.5 using HCl (2 M), and centrifuged at 3000 rpm for 25 minutes. Samples were washed twice using pure water and quantified. Around 0.2 mL solution containing alcalase (0.05%) and inhibitor solution (protein) was incubated with potassium phosphate buffer (0.1 M) having pH 8.0 for 6 hours at 37°C. To stop the hydrolysis, samples were boiled for 6-7 min and centrifuged at room temp for 10-15 minutes [24].

### 2.5. Characterization of Peptides

#### 2.5.1. SDS-PAGE Analysis of ACE Inhibitory Peptides

SDS-PAGE was used for the determination of the molecular mass of hydrolyzed proteins. Hydrolyzed proteins were dissolved in a buffer containing SDS and separated on a polyacrylamide gel matrix. After electrophoresis, the gel was carefully removed and placed in Coomassie blue staining solution for 1 hour [25]. The gel was destained for 60 minutes, and the bands were compared with a standard protein marker to determine the molecular mass of hydrolyzed proteins of cottonseeds, peanuts, and chickpeas.

#### 2.5.2. LC-MS/MS Analysis of Peptides

The hydrolyzed peptide fraction was introduced into a mass spectrometer (ISQ™ EM Single Quadrupole Mass Spectrometer, ISQEM-ESI-APCI, Thermo Fisher Scientific, Germany) using an electrospray ionization source. The spectra were obtained with a mass range of 50-2000 *m*/*z* in positive ionization mode. MS/MS was operated at 4.0 kV spray voltage, auxiliary gas 5 units/min, sheath gas 15 unit/min, 275°C capillary temperatures, and 100.50 V tube voltage. The fragmentation was carried out with collision-induced dissociation (CID) of 25-30 units/mass. The spectral data of ion peaks were obtained using Xcalibur Software (Thermo Fisher Scientific™).

RETRACTED

### 2.6. Statistical analysis

All samples used in this study were measured as an average of triplicates. The data collected were analyzed by computing standard errors [26].

## 3. Results and Discussion

### 3.1. ACE Inhibitory Activity of Plants

Cottonseeds showed maximum ACE inhibitory activity (55%), followed by peanut (50%), chickpea (47%), papaya seeds (36.5%), and flaxseed (31%) (Figure 1). The variation in ACE interdict potential may be due to the different plant types and the nature of protein present in plants, or it may be ascribed as the presence of other metabolites in the extract which may interfere with the inhibition activity [27].

### 3.2. Effect of pH, Temperature, Hydrolysis Time, and Enzyme to Substrate (E/S) Ratio on ACE Inhibition (%) Activity

Extremely high or low pH may completely result in the loss of activity of enzymes [28]. The effect of different pH (6-9) on ACE inhibition (%) of cottonseed, peanut, and chickpea was studied. Our study showed that change in pH significantly affected the ACE inhibition (%). By increasing pH, ACE inhibitory (%) action of cottonseed, peanut, and chickpea was augmented. An increase in pH from 6.0 to 8.0 resulted in the more ACE inhibitory activity of cotton seed (77%), peanut (76%), and chickpea (48%) proteins (Figure 2(a)). Cottonseed and peanut showed maximum ACE inhibition activity at pH 8.0 while chickpea at pH 7.0 (Figure 2(b)). Previous studies reported that optimum pH level is different for different plants and dependent upon reaction conditions [29].

Our studies demonstrate that a gradual increase in temperature resulted in increased ACE inhibition activity of cottonseed, peanut, and chickpea. The rise in temperature from 35 to 45°C resulted in increased ACE activity from 18% to 77.5% for cottonseed (Figure 2(a)) and 76.1% for peanut (Figure 2(b)). Chickpea protein showed increased ACE activity from 26% to 46% with increasing pH (Figure 2(c)). Our study disclosed that a rise in temperature led to 45°C increased ACE inhibition activity (10% to 70%) in cottonseed and peanut (Figures 3(a) and 3(b)), whereas increasing the temperature to 40°C decreased (48% to 33%) the ACE inhibitory activity in chickpea protein (Figure 3(c)). According to the enzymatic reaction dynamic principle, by increasing temperature, the reaction rate also increases, but here, this decrease in enzyme activity can be described as most of the enzyme denature as temperature increases to 40°C or even higher [30]. Previous studies proved that increase in temperature above the optimum temperature did not result in higher inhibition activity and also inhibits the hydrolysis reaction [31] which best supports our study results.

RETRACTED

Our study results disclosed that cottonseed, peanut, and chickpea proteins showed maximum ACE inhibitory action when the hydrolysis reaction was performed for 2 hours (Figures 4(a)–4(c)). After 2 hrs hydrolysis time, chickpea, peanut, and cottonseed showed 46% (Figure 4(a)), 45% (Figure 4(b)), and 69% (Figure 4(c)) ACE inhibition activity, respectively. An increase in hydrolysis reaction time to 8 hrs resulted in gradually reduced ACE inhibition activity. Our study results are best supported by earlier findings [32]. An increase in time above 2 hrs did not cause any positive effect on protein yield and terminated the hydrolysis reaction [33].

The enzyme to substrate (E/S) ratio plays an important role in protein hydrolysis. It is clear from the experiments that if the concentration of enzymes is kept constant and the amount of substrate is increased then the rate of forwarding reaction enhances but only at a specific value because a further increase in E/S decreases the rate of reaction. Different E/S ratios were analyzed on cottonseed, peanut, and chickpea, i.e., from 1 : 3 to 1 : 9 under similar reaction conditions. We found that an increase in enzyme to substrate ratio resulted in increased ACE suppression activity. Cottonseed showed maximum ACE inhibitory activity (86%) at 1 : 5 (Figure 5(a)), peanut (68%) at 1 : 7 (Figure 5(b)), and chickpea (70%) at 1 : 9 E/S ratio (Figure 5(c)). Previous findings also reported that increased enzyme to substrate ratio resulted in increased turnover of protein hydrolysates [34, 35] which best supports our findings.

### 3.3. Polyacrylamide Gel Electrophoresis (SDS-PAGE)

Our results demonstrated the molecular weight of cottonseed protein fraction of 39 kDa while chickpea protein showed 25 kDa and 150 kDa subunits, which indicate the presence of vicilin subunit of electrophoresed protein (Figure 6). Our study findings revealed that the molecular weight of peanut protein fractions of 20 kDa, 55 kDa, and 150 kDa (Figure 6) can be recognized as cruciferin and napin subunits of hydrolyzed protein [36]. Therefore, it is revealed from SDS-PAGE that hydrolysis with alcalase enzyme is important for the production of smaller subunits of protein that can be valuable candidates for antihypertensive treatment.

RETRACTED

### 3.4. LC-MS/MS Analysis of Peptides

Liquid chromatography mass spectrometry (LC-MS/MS) is a powerful analytical technique, used for the identification of unknown compounds, and structure elucidation to find the chemical properties of different compounds/peptides. It is highly sensitive and selective for the analysis of compounds present in trace amounts [37, 38]. In the current study, LC-MS/MS is used for identification and structure elucidation of bioactive peptides to find the sequence of peptides present in a hydrolyzed fraction of cottonseed plant, i.e., Valine-Glycine (Val-Gly), Serine-Threonine (Ser-Thr), Histidine-Threonine (His-Thr), Glycine-Glycine-Histidine (Gly-His-His), Phenylalanine-Methionine (Phe-Met), Valine-Proline-Glycine-Glycine (Val-Pro-Gly-Gly), Lysine-Valine-Tryptophan (Lys-Val-Trp), and pentapeptide Glutamic acid-Glycine-Alanine-Serine-Aspartic acid (Glu-Gly-Ala-Ser-Asp) (Table 1). LC-MS/MS analysis of hydrolyzed fraction obtained from cotton seed showed peptides in positive ionization mode. The molecular peak at *m*/*z* 146 [M+H]^+^ in the mass spectrum (Figure 7) was identified as valine-glycine dipeptide which showed other ions at *m*/*z* 56.75 due to [M+H-Val] and *m*/*z* 73.83 due to removal of [valine-NH=CH] in fragmentation pattern specific for Val-Gly dipeptide. The fragment ion spectra in our study were in agreement with the fragment ion peaks of Val-Gly peptide as reported earlier in plants [39, 40]. The peak at *m*/*z* 189 identified as Ser-Thr [M+H]^+^ (Figure 7). Pattern visualized at *m*/*z* 101.92 is due to the removal of threonine [M+H-Thr], at *m*/*z* 71.83 by dehydration [Ser-H_2_O], and at *m*/*z* 72.33 due to the elimination of [Thr-NH=CH]. Molecular ion peak at *m*/*z* 239 [M+H]^+^ was detected as His-Thr dipeptide, at *m*/*z* 193.17 due to the removal of [M+H-45], and *m*/*z* 157.75 due to the removal of [M+H-81] (Figure 7).

The peak at *m*/*z* 253 [M + H]^+^ corresponds to the His-Gly-Gly tri-peptide. The product peak at *m*/*z* 137.92 due to the [M + H-Gly-Gly] and at *m*/*z* 109.83 due to [His-NH=CH], and *m*/*z* 120 due to the removal of [His-H_2_O]. A molecular ion peak at *m*/*z* 280 [M+H]^+^ was identified as Phe-Met dipeptide (Figure 7) which produced a minor band at *m*/*z* 148.83 due to the phenylalanine amino acid, at *m*/*z* 166.92 due to the addition of water molecule [Phe+H_2_O], at *m*/*z* 133.92 due to the methionine amino acid, and at *m*/*z* 115.92 due to dehydration [Met-H_2_O] (Figure 7). The fragment ion profile in our study was similar to that reported previously [37]. The precursor ion at *m*/*z* 312 [M+H]^+^ was detected as Val-Pro-Gly-Gly tetra-peptide. Spectra produced at *m*/*z* 255.83 and *m*/*z* 197.00 resulted due to the elimination of [M+H-Gly-Gly], *m*/*z* 213.02 due to the [M+H-Pro], and *m*/*z* 100.83 due to the Val peptide (Figure 7). A molecular ion peak at *m*/*z* 413 [M+H]^+^ was due to Lys-Val-Trp tripeptide (Figure 7), which produced peaks at *m*/*z* 314.18 due to [M+H-Val], *m*/*z* 369.1 due to [M+H-43], and *m*/*z* 338.6 due to [M+H-73], and 226.00 is ascribed due to [M+H-Trp]. Pentapeptide Glu-Gly-Ala-Ser-Asp produced ion spectrum band at *m*/*z* 459 [M+H]^+^, spectra at *m*/*z* 360.33 due to [M+H-Val], *m*/*z* 441.16 due to dehydration [M+H-H_2_O], *m*/*z* 429.34 due to [M+H-31], *m*/*z* 401.00 due to [M+H-58], and *m*/*z* at 344.17 in the spectra can be attributed due to [M+H-Asp] (Figure 7). Previous studies have reported that peptides having different amino acid sequences possess different ACE inhibition activities [41–44]. Further exploration of the multiple and different peptides of these cottonseed proteins may shed more light on the evolution, posttranslational modification, and isoform of cottonseed and other plant proteins with the potential of ACE inhibitory candidate peptides. The further in-depth study could also provide novel insight into the functional utilization of the relevant bioactive peptide fragments to determine whether they are the peptide precursors or the degraded product.

RETRACTED

## 4. Conclusion and Future Outlook

According to the best of our information available, this was the first performed study regarding the protein profiling of cottonseed using LC-MS/MS technique, and the peptides obtained are explored for the first time. From the current findings, it is clear that cottonseed, peanut, and chickpea have the potential against hypertension. However, among all the studied plants, cottonseed contains important amino acids which are essential for antihypertensive activity. Hence, it can be concluded that antihypertensive proteins from cottonseed are valuable alternatives because of their cost-effectiveness and no side effect.

### 4.1. Study Limitations/Recommendations

There must be detailed studies on the specific structural unit of the peptides by MALDI-TOF analysis, which is very costly and time taking, followed by docking analysis and protein-protein interactions to analyze the best fit model of peptides in autoimmune disorders/diseases.

## Figures and Tables

**Figure 1:** ACE inhibition activity of plant seed extracts.

**Figure 2:** (a) Optimization of pH for hydrolysis of cotton seed proteins. (b) Optimization of pH for hydrolysis of peanut proteins. (c) Optimization of pH for hydrolysis of chickpea proteins.

RETRACTED

**Figure 3:** (a) Optimization of temperature for hydrolysis of cottonseed protein. (b) Optimization of temperature for hydrolysis of peanut protein. (c) Optimization of temperature for hydrolysis of chickpea protein.

**Figure 4:** (a) Optimization of time for hydrolysis of chickpea protein. (b) Optimization of time for hydrolysis of peanut protein. (c) Optimization of time for hydrolysis of cottonseed protein.

**Figure 5:** (a) Optimization of E/S for hydrolysis of cottonseed protein. (b) Optimization of E/S for hydrolysis of peanut protein. (c) Optimization of E/S for hydrolysis of chickpea protein.

**Figure 6:** SDS-PAGE results for hydrolysis cottonseed, chickpea, and peanut proteins.

**Figure 7:** LC-MS/MS spectrum of hydrolyzed cottonseed protein.

**Table 1:** Peptides identified in hydrolyzed protein profile of cottonseed in positive ionization mode.

Peptide	Peptide structure
Valine-Glycine (Val-Gly)	
Serine-Threonine (Ser-Thr)	
Histidine-Threonine (His-Thr)	
Glycine-Glycine-Histidine (Gly-His-His)	
Phenylalanine-Methionine (Phe-Met)	
Valine-Proline-Glycine-Glycine (Val-Pro-Gly-Gly)	
Lysine-Valine-Tryptophan (Lys-Val-Trp)	
Glutamic acid-Glycine-Alanine-Serine-Aspartic acid (Glu-Gly-Ala-Ser-Asp)	

## Data Availability

All the data relevant to this study are mentioned in the manuscript. There are no any supplementary data.
